The article "Prognostic Value of an Integrin-Based Signature in Hepatocellular Carcinoma and the Identification of Immunological Role of LIMS2" was published in 2022. Journal: Dis Markers.

# Prognostic Value of an Integrin-Based Signature in Hepatocellular Carcinoma and the Identification of Immunological Role of LIMS2

**DOI:** 10.1155/2022/7356297

**Published:** 2022-09-29

**Authors:** Fengning Ye, Hao Le, Fan He, Hao Tu, Dengfa Peng, Sini Ruan

**Affiliations:** ^1^Ultrasound Imaging Department, The National Hospital of Enshi Autonomous Prefecture, Enshi, China; ^2^First Surgical Department, The National Hospital of Enshi Autonomous Prefecture, Enshi, China; ^3^Ultrasound Imaging Department I, The Central Hospital of Enshi Tujia and Miao Autonomous Prefecture, Enshi, China

## Abstract

**Objective:**

Evidence proves that integrins affect almost every step of hepatocellular carcinoma (HCC) progression. The current study aimed at constructing an integrin-based signature for prognostic prediction of HCC.

**Methods:**

TCGA-LIHC and ICGC-LIRI-JP cohorts were retrospectively analyzed. Integrin genes were analyzed via univariate Cox regression, followed by generation of a prognostic signature with LASSO approach. Independent factors were input into the nomogram. WGCNA was adopted to select this signature-specific genes. Gene Ontology (GO) enrichment together with Kyoto Encyclopedia of Genes and Genomes (KEGG) pathway analysis were conducted to explore the function of the dysregulated genes. The abundance of tumor microenvironment components was estimated with diverse popular computational methods. The relative importance of genes from this signature was estimated through random-forest method.

**Results:**

Eight integrin genes (ADAM15, CDC42, DAB2, ITGB1BP1, ITGB5, KIF14, LIMS2, and SELP) were adopted to define an integrin-based signature. Each patient was assigned the riskScore. High-riskScore subpopulation exhibited worse overall survival, with satisfying prediction efficacy. Also, the integrin-based signature was independent of routine clinicopathological parameters. The nomogram (comprising integrin-based signature, and stage) accurately inferred prognostic outcome, with the excellent net benefit. Genes with the strongest positive interaction to low-riskScore were primarily linked to biosynthetic, metabolic, and catabolic processes and immune pathways; those with the strongest association with high-riskScore were principally associated with diverse tumorigenic signaling. The integrin-based signature was strongly linked with tumor microenvironment components. Among the genes from this signature, LIMS2 possessed the highest importance, and its expression was proven through immunohistochemical staining.

**Conclusion:**

Altogether, our study defined a quantitative integrin-based signature that reliably assessed HCC prognosis and tumor microenvironment features, which possessed the potential as a tool for prognostic prediction.

## 1. Introduction

Liver cancer remains the sixth most commonly diagnosed cancer together with the third most deadly cancer, with an estimated 906,000 new cases as well as 830,000 deaths globally [1]. Asian countries have the highest incidence of primary liver cancer cases, reporting approximately 72.5% of the world's cases [2]. Hepatocellular carcinoma (HCC) contributes 80% of all cases worldwide [3]. Elderly male together with Asian populations are still the highest risk groups for HCC. The preferred therapy of HCC remains surgery, which is the only method to achieve long-term survival and even a cure [4]. Radiofrequency ablation is the treatment of choice for malignancies that are extremely early in their stages as well as tumors that are early in their stages but cannot be removed surgically [5]. Ultrasound is well poised to address this need due to its low cost, portability, safety, and excellent temporal resolution. The role of ultrasound for HCC screening has been well established and supported by multiple international guidelines. Nonetheless, HCC patients are generally in intermediate or advanced stages. Transcatheter arterial chemoembolization is the standard of care for patients with intermediate HCC, resulting to the median survival of 25–30 months [6]. Molecular-targeted agents, sorafenib, etc. have been developed against advanced HCC [7]. Regrettably, liver toxicity and weak anti-tumor effect contribute to treatment failure and low survival benefit. Recently, immune-based therapies have generated notable improvement in clinical outcome of HCC [8]. Despite this, current immunotherapies only induce durable response for minority of HCC patients. Altogether, it is of significance to select potent therapeutic targets, and determine more reliable tools for stratifying HCC patients together with prognostic prediction.

Integrins cross the plasma membrane as well as connect the extracellular matrix (ECM) to the cytoskeleton, as elementary cell adhesion receptors mediating cellular and tissue functions [9]. Altered expression of integrins is commonly detected in HCC [10]. They profoundly affect almost every step of HCC progression from primary tumor development to metastases [10, 11]. Additionally, integrins correlate to the acquisition of drug resistance and immune escape [12, 13]. In addition to tumor cells, integrins are present in components within tumor microenvironment, which critically regulate their contributions to tumor progression [14]. For instance, SPON2 facilitated the recruitment of M1-like macrophages as well as mitigates HCC metastases through integrin signaling [10]. Cancer-associated fibroblasts facilitate vascular invasion of HCC through lowering integrin *β*1 [15]. Blockade of integrin signaling can attenuate HCC progression through hindering key signaling events in tumor microenvironment and tumor cells. Hence, integrins together with integrin-dependent functions have been regarded as attractive therapeutic targets against HCC [16]. In addition to this, integrins may become imaging biomarkers for evaluating the efficacy of anti-angiogenic or anti-tumor agents [17]. Moreover, integrin-targeted nanoparticles with varying anti-tumoral payloads are a definitely promising research field to lower toxicity linked to systemic radio- or chemotherapy [18]. To date, the now prognostic model based on integrin-related genes were rarely reported. Based on accumulated evidence, the current study conducted a comprehensive analysis of multidimensional integrin-relevant genomic data across HCC, and defined a quantitative integrin-based signature that may evaluate HCC prognostic outcome together with tumor microenvironment traits, which might open up a novel insight into improving HCC outcomes together with determining patients' therapeutic regimens.

## 2. Materials and Methods

### 2.1. Data Acquisition

Transcriptome data and clinical information of HCC patients were acquired from TCGA-LIHC as the training cohort. Under removal of patients with incomplete survival data, 343 HCC patients were included. Another RNA-seq dataset ICGC-LIRI-JP with 229 HCC samples obtained from the ICGC database were adopted for verification.

### 2.2. Collection of Integrin Gene Set

The Molecular Signatures Database offers the annotated gene sets that involve biochemical pathways, signaling cascades, and expression profiling from published research together with other biological concepts [19]. We collected 128 integrin genes from this popular database, involving four biological process terms (integrin activation, integrin-mediated signaling pathway, positive regulation of integrin activation, and regulation of integrin activation) together with one cellular component terms (integrin complex).

### 2.3. Definition of an Integrin-Based Signature

Prognostic significance of integrin genes was firstly evaluated. Through adopting univariate-cox regression approach, integrin genes with *p* < 0.05 were selected, and input into least absolute shrinkage and selection operator (LASSO) [20]. This analysis was conducted utilizing glmnet package [21]. The regression coefficient was computed utilizing multivariate-cox regression. The integrin-based signature-derived riskScore was generated through combination of regression coefficient together with transcript level of each integrin gene in this signature. With the median riskScore, patients were classified as low- and high-riskScore subpopulations. This classification was verified through PCA and tSNE approaches. Overall survival (OS) analysis was implemented with Kaplan–Meier (K-M) method together with log-rank test. Area under the receiver operating characteristic curve (AUC) was computed with “timeROC” package. Uni- together with multivariate-cox regression methods were adopted for inferring the independency of the integrin-based signature as a prognostic parameter. Through the use of subgroup analysis, we were able to deduce the sensitivity of this signature in prognostic prediction.

### 2.4. Nomogram Construction

Nomogram was generated through incorporating independent risky factors (riskScore and stage) via adopting rms package. ROC curves were utilized for reflecting the predictive capability of the nomogram. Concordance index (C-index) was employed to estimate the nomogram discrimination through bootstrap approach with 1000 resamples. Calibration curve was graphically assessed through drawing the actual OS rate against the probability predicted by this nomogram, with the 45° line for the ideal prediction. Decision curve analysis was employed to evaluate the net benefit of the nomogram, routine clinicopathological parameters, and riskScore.

### 2.5. Weighted Gene Coexpression Network Analysis (WGCNA)

WGCNA package [22] was adopted to select the riskScore-specific modules. The transcriptome profiling was utilized as input for WGCNA, and riskScore was computed as well as defined as the clinical traits. A signed scale-free coexpression gene network was guaranteed via setting an appropriate power *β* value and scale-free *R*^2^ value as the soft threshold parameters. Afterwards, we constructed a coexpression matrix in accordance with *β* value, and the input gene expression matrix for classifying genes with similar expression pattern into the same gene module, thus producing a coexpression module. Association of module Eigengenes with riskScore were estimated with Eigengenes function. Heatmap was generated for visualizing the association of each coexpression module with riskScore. Modules with the strongest association with riskScore were selected as the riskScore-specific modules.

### 2.6. Functional Enrichment Analysis

Gene Ontology (GO) enrichment together with Kyoto Encyclopedia of Genes and Genomes (KEGG) pathway analysis were conducted through adopting clusterProfiler package [23]. For preventing high false discovery rate (FDR) in multiple tests, *q*-value was inferred for FDR control. A gene set was regarded as significantly enriched if a *p* < 0.05 and false discovery rate <0.025.

### 2.7. Estimation of Tumor Microenvironment Components

Seven computational approaches were employed to infer components within tumor microenvironment. Tumor Immune Estimation Resource (TIMER) adopts deconvolution approach to estimate the level of six tumor-infiltrating immune subsets from gene expression profiling [24]. CIBERSORT applies transcriptome profiles with a predefined immune signature matrix to calculate the deconvolution of 22 tumor-infiltrating immune cells in a given sample on the basis of support-vector regression [25]. quantTIseq quantifies the fraction of 10 immune cell types utilizing bulk RNA-sequencing data [26]. MCPcounter quantifies the absolute abundance of 8 immune together with 2 stromal cell subsets within heterogeneous tissues through transcriptomic profiles [27]. XCELL infers 64 immune, and stromal cell types via adopting gene signature-based approach [28]. EPIC estimates the proportion of immune and cancer cells utilizing bulk gene expression profiling [29]. Associations of riskScore and genes in the integrin-based signature with the abundance of tumor microenvironment components were estimated with Spearman's correlation test.

### 2.8. Random-Forest Analysis

The relative importance of genes in the integrin-based signature was ranked via implementing random-forest analysis, and the gene with the highest importance was determined. LIMS2 transcript level was compared between low- and high-riskScore subpopulations. Association of LIMS2 transcript level with riskScore was inferred with Spearman's correlation test. Immunohistochemical staining of LIMS2 in HCC and normal tissue was acquired from the Human Protein Atlas.

#### 2.8.1. Patients and Tissue Samples

The study was approved by the Ethic Committee of The National Hospital of Enshi Autonomous Prefecture. Written informed consent on the use of clinical specimens from each patient was achieved. Eight pairs of HCC tissues and matched nontumor tissues were acquired from HCC patients with written informed consents who received surgical resection at The National Hospital of Enshi Autonomous Prefecture. These tissue samples were confirmed by pathological diagnoses and stored at -80°C until use.

#### 2.8.2. RT-qPCR

Total RNA from HCC specimens and nontumor specimens was extracted by the use of the TRIzol kit (Invitrogen, China). A reverse transcription kit was applied to synthesize the cDNA. Based on the instructions of the SYBR Premix Ex Taq kit (Takara, Dalian, China), Real-time PCR experiments were carried out. The relative quantification of genes was assessed using the 2^−∆∆Ct^ method. The primer sequences were presented as follows: LIMS2 5′-GCACCGGCACTATGAGAAGAA-3′ (forward) and 5′-ACGGGCTTCATGTCGAACTC-3′ (reverse), GAPDH 5′-GCCACATCGCTCAGACACCAT-3′, and 5′-CCCATACGACTGCAAAGACCC-3′.

### 2.9. Statistical Analysis

All statistical tests were conducted with R software (R Statistical Software, R Foundation for Statistical Computing, Vienna, Austria). *p* < 0.05 indicated statistical significance.

## 3. Results

### 3.1. Definition of an Integrin-Based Signature for HCC Prognostic Outcome

To observe the prognostic signature of integrin genes, the current study carried out univariate-cox regression analysis in TCGA-LIHC cohort. Among 128 integrin genes, 35 exhibited significant correlations to OS (Figure 1(a)). Among them, FBLN1, FLNA, ITGB1, ITGA3, LAMA5, CDH17, SRC, COL16A1, ITGA2, ZYX, ITGAM, ITGAV, NME2, ABL1, CD63, ILK, PTGER4, PRKD1, ADAM9, PTK2, ITGA5, DAB2, ADAM15, BCAR1, ITGB5, LIMS1, RCC2, CTNNA1, ITGB1BP1, KIF14, RAP1B, and CDC42 act as risky factors, with LIMS2, SELP, and APOA1 as protective factors. These prognostic integrin genes were adopted for defining an integrin-based signature with LASSO approach (Figures 1(b) and 1(c)). The formula of the integrin-based signature was as follows: riskScore = 0.0827089185245466, ^∗^ADAM15 transcript level + 0.0709032023435198, ^∗^CDC42 transcript level + 0.128150636135253, ^∗^DAB2 transcript level + 0.196471754226477, ^∗^ITGB1BP1 transcript level + 0.121662581037157, ^∗^ITGB5 transcript level + 0.207623740869238, ^∗^KIF14 transcript level + (−0.31147424622991), ^∗^LIMS2 transcript level + (−0.0983574871616035), and ^∗^SELP transcript level (Figure 1(d)). With K-M curve together with log-rank test, the prognostic implication of each gene in integrin-based signature was further verified across TCGA-LIHC. Consequently, highly expressed SELP and LIMS2 correlated to more favorable OS, with highly expressed KIF14, ITGB5, DAB2, CDC42, ADAM15, and ITGB1BP1 linked to poorer OS (Figures 1(e)–1(l)).

### 3.2. The Integrin-Based Signature Excellently Predicts HCC's OS Outcome

We stratified TCGA-LIHC together with ICGC-LIRI-JP cases into low- and high-riskScore subpopulations following the median riskScore (Figures 2(a) and 2(b)). Both in two cohorts, more dead cases were observed in high-riskScore subpopulation (Figures 2(c) and 2(d)). ADAM15, CDC42, DAB2, ITGB1BP1, ITGB5, and KIF14 displayed higher transcript level in high- than low-riskScore subpopulation, with lower transcript level of SELP, and LIMS2 in high-riskScore subpopulation across TCGA-LIHC as well as ICGC-LIRI-JP cases (Figures 2(e) and 2(f)).

Afterwards, OS outcome was compared between subpopulations across TCGA-LIHC. In contrast to high-riskScore patients, those with low-riskScore possessed the notable advantage in OS outcome (Figure 3(a)). ROC curves were plotted to investigate the prediction efficacy of the integrin-based signature. Consequently, AUC values of OS at one, two together with three years were all exceeding 0.7 (Figure 3(b)), proving that this signature excellently predicted HCC's OS outcome. To verify the discrepancy between low- and high-riskScore subpopulations, we adopted PCA and tSNE approaches across TCGA-LIHC. As a result, low-riskScore patients signally distinguished from those with high-riskScore at the transcriptome level (Figures 3(c) and 3(d)).

Next, the current study observed whether the integrin-based signature generalized to other cohorts. Similarly, we computed riskScore of patients from ICGC-LIRI-JP cohort, which were then classified as low- and high-riskScore subpopulations. As expected, poorer OS outcome was proven in high-riskScore subpopulation (Figure 3(e)). In addition, AUC values of OS at one, two together with three years were all over 0.7 (Figure 3(f)). PCA and tSNE demonstrated the arresting discrepancy between subpopulations (Figures 3(g) and 3(h)).

The integrin-based signature is independent of routine clinicopathological parameters.

Next, the present study estimated the associations of riskScore and routine clinicopathological parameters with OS outcome across TCGA-LIHC utilizing univariate-cox regression approach. Consequently, riskScore together with stage were linked with poor OS outcome (Figure 4(a)). Multivariate-cox regression approach was adopted to infer whether riskScore was independent of routine clinicopathological parameters. As illustrated in Figure 4(b), riskScore together with stage acted as independent risky factors of TCGA-LIHC. The sensitivity of riskScore in prognosis prediction was measured in diverse subgroups stratified by routine clinicopathological parameters (sex, grade, or stage). In each subgroup, high-riskScore subpopulation possessed worse OS outcome in contrast to low-riskScore subpopulation (Figures 4(c)–4(h)).

### 3.3. Generation of an Integrin-Based Signature- and Stage-Based Nomogram into HCC Clinical Practice

Two independent risky factors (riskScore together with stage) were selected for generating a nomogram for HCC prognostic prediction (Figure 5(a)). Firstly, points for riskScore and stage were derived in TCGA-LIHC cases. Total points were acquired through adding the points of two risky factors, and the corresponding location of the point of each patient was observed in the line of total points. At last, the probability of one-, three- together with five-year OS for HCC was referred through plotting a straight line on the bottom three rows. ROC curves and C-indices were adopted for evaluating the prediction accuracy of the nomogram. AUC values of OS at one, two together with three years were all over 0.7 (Figure 5(b)), and the C-indices were over 0.7 for short- and long-term OS outcomes (Figure 5(c)). In addition, calibration curve illustrated that the one-, three- together with five-year OS probability predicted by this nomogram was consistent with the actual OS rate (Figure 5(d)). Above evidence proved the excellent prediction efficacy of this nomogram. Decision curve analysis curves at one-, three- together with five-year OS displayed the potential for clinical application as well as better net benefits (Figures 5(e)–5(g)).

### 3.4. Selection of Integrin-Based Signature-Specific Genes

WGCNA was employed for identifying integrin-based signature-specific genes across TCGA-LIHC. Transcriptome data and clinical trait (low- and high-riskScore) were input into WGNCA. The first power value when the index of scale-free topologies was up to 0.90 was set as the optimal soft threshold power (*β*) for establishing a scale-free network, and genes with similar expression patterns were assigned to the same coexpression module utilizing dynamic tree cut approach, thus generating 12 coexpression modules (Figures 6(a)–6(c)). Afterwards, associations of coexpression modules with low- and high-riskScore were evaluated. Turquoise module exhibited the strongest positive interaction to low-riskScore (Figure 6(d)). In addition, yellow module displayed the strongest positive association with high-riskScore. Thus, genes in turquoise and yellow modules were regarded as integrin-based signature-specific genes.

Next, biological implication of integrin-based signature-specific genes was assessed. Genes in turquoise module were primarily linked to biosynthetic, metabolic, and catabolic processes together with immune pathways (Figures 6(e) and 6(f)). Genes in yellow module primarily correlated to diverse tumorigenic signaling (Figures 6(g) and 6(h)).

### 3.5. Interactions of the Integrin-Based Signature with Components within Tumor Microenvironment

Diverse computational approaches were adopted for inferring the interactions of the integrin-based signature with components within tumor microenvironment across TCGA-LIHC. Overall, high-riskScore exhibited higher abundance of immunosuppressive cells, and the riskScore was positively correlated to immunosuppressive cells (Figures 7(a) and 7(b)). In addition, genes from the integrin-based signature (ADAM15, CDC42, DAB2, ITGB1BP1, ITGB5, KIF14, SELP, and LIMS2) were strongly linked with the abundance of components within tumor microenvironment (Figures 7(c)–7(i)).

### 3.6. The Importance of LIMS2 from the Integrin-Based Signature in HCC

Random-forest approach was adopting for assessing the relative importance of genes in the integrin-based signature. Consequently, LIMS2 possessed the highest importance (Figure 8(a)). In contrast to low-riskScore subpopulation, lower transcript level of LIMS2 was observed in high-riskScore subpopulation (Figure 8(b)). In addition, LIMS2 transcript level was negatively linked to riskScore (Figure 8(c)). Immunohistochemical staining demonstrated that LIMS2 protein displayed low expression level in normal tissue, without detection in HCC tissue (Figures 8(d) and 8(e)). Finally, we performed RT-PCR and found that LIMS2 expression was distinctly decreased in HCC specimens compared with nontumor specimens (Figure 8(f)).

## 4. Discussion

Despite the notable improvement in HCC research, patients' outcome remains depressing [30]. Hence, it is imperative to search for novel tools for HCC prognostic prediction. Evidence demonstrates that integrins affect almost every step of HCC progression [10]. Herein, eight integrin genes (ADAM15, CDC42, DAB2, ITGB1BP1, ITGB5, KIF14, LIMS2, and SELP) were selected and adopted to define an integrin-based signature. High-riskScore subpopulation displayed worse OS, with satisfying prediction efficacy. In addition, the integrin-based signature was independent of routine clinicopathological parameters. To facilitate clinical practice, we produced the integrin-based signature- and stage-based nomogram that accurately inferred prognostic outcome, with the excellent net benefit.

Accumulated evidence proves the significance of genes from the integrin-based signature in HCC. For instance, ADAM15 metalloproteinase, a multidomain disintegrin protease, is linked to prognostic outcome, infiltration of immune cells together with apoptosis in HCC [31]. CDC42 stimulates tumor growth, angiogenesis together with metastatic potential of HCC [32]. DAB2 mitigates tumor growth and metastasis of HCC [33]. ITGB1BP1 induces HCC metastasis through epithelial-mesenchymal transition [34]. ITGB5 motivates HCC tumorigenesis via elevating *β*-catenin stability [35]. KIF14 suppression may interfere with cell cycle progression together with cytokinesis through hindering p27 ubiquitination signaling in HCC [36]. In addition, KIF14 expedites growth and sorafenib resistance in HCC [37]. Microwave responsive nanoplatform through SELP-mediated drug delivery exhibits the excellent efficacy in treating HCC with distant metastasis [38].

To unveil the mechanisms underlying the integrin-based signature-derived riskScore, specific genes were selected, respectively. Genes with the strongest positive interaction to low-riskScore were primarily correlated to biosynthetic, metabolic, and catabolic processes and immune pathways. In addition, genes with the strongest association with high-riskScore were principally linked with diverse tumorigenic signaling. Above data reflected the prognostic difference between low- and high-riskScore subpopulations. Tumorigenesis-related inflammation results in the accumulation of immune cells within tumors together with the surrounding environment, which contributed to tissue remodeling as well as damage in their functions [39]. Immune cells and nonimmune components comprise the immediate surrounding of tumor cells, named tumor microenvironment [40]. Components within tumor microenvironment exert dual roles in HCC. Tumor microenvironment was in charge of immune surveillance together with immunoediting [41]. In addition, it facilitates invasive tumor growth, metastatic potential as well as evasion from immune surveillance [42]. The current evidence proved the interactions of the integrin-based signature and their genes with tumor microenvironment components across HCC.

Among genes from the integrin-based signature, LIMS2 possessed the highest importance. LIMS2 was negatively linked with riskScore and exhibited low expression in HCC. Additionally, its expression in HCC was proven via immunohistochemical staining. Previously, LIMS2 inhibition contributed to enlargement of liver and tumorigenesis [43]. Epigenetic silencing of LIMS2 has been found in gastric cancer [44]. Extracellular vesicles secreted by mesenchymal stem cells inhibit the progression of cervical cancer by transferring the microRNA miR-331-3p, which reduces the level of methylation of LIMS2 in cancer cells [45]. Our study presented for the first time the importance of LIMS2 in HCC. LIMS2 might become a potent therapeutic target of HCC.

Nonetheless, this study has a few disadvantages. Firstly, we utilized the LASSO approach to filter prognostic integrin genes. Regrettably, the disadvantages of this approach itself possibly resulted in missing some integrin genes with equally important contributions when adjusting the regression coefficients. In addition, clinical features incorporated in the independent analysis of the prognostic signature together with the establishment of the nomogram were traditionally considered crucial factors influencing HCC tumorigenesis. Nonetheless, a few clinical elements with similar contributions, dietary habits, etc., were not incorporated in our study as a result of insufficient patients' information, which might impact our conclusions. In addition, the efficacy of the prognostic signature used to assess immunotherapeutic response will be further proven in large clinical trials.

## 5. Conclusion

In summary, the integrin-based signature was generated and verified, which possessed predictive significance of HCC prognostic outcome. Our findings supported the notions that integrin genes notably correlated to patients' outcome. In clinical practice, to measure the transcript level of only ADAM15, CDC42, DAB2, ITGB1BP1, ITGB5, KIF14, LIMS2, and SELP might be a cost-effective application and enabled to offer accurate prognostic prediction of HCC.

## Figures and Tables

**Figure 1:** Definition of an integrin-based signature for HCC prognostic outcome in TCGA-LIHC cohort. (a) Forest diagram illustrates the significant correlations of 35 integrin genes with HCC OS. Red, risky factor; and green, protective factor. (b) LASSO coefficient profiling of 35 prognostic integrin genes describes that the alterations in the magnitude of the variable coefficients shrinks as the penalty value increases. (c) Penalty diagram shows the partial likelihood deviance under diverse penalty values. (d) The coefficient of each gene in the integrin-based signature. (e–l) K-M curves of OS outcomes between highly and lowly expressed SELP, LIMS2, KIF14, ITGB5, DAB2, CDC42, ADAM15, or ITGB1BP1 groups. OS difference was estimated with log-rank test.

**Figure 2:** Calculation of the integrin-based signature-derived riskScore in TCGA-LIHC together with ICGC-LIRI-JP cohorts. (a) Distribution of riskScore across TCGA-LIHC cases. Vertical dashed line denotes the median riskScore. TCGA-LIHC cases are classified as low- and high-riskScore subpopulations. (b) Distribution of riskScore across ICGC-LIRI-JP cases. (c) Survival time and status across TCGA-LIHC cases with increasing riskScore. Blue, alive; red, dead. (d) Survival time and status across ICGC-LIRI-JP cases with increasing riskScore. (e) Heatmap visualizes transcript level of genes in the integrin-based signature across low- and high-riskScore subpopulations from TCGA-LIHC cohort. Blue, low transcript level; red, high transcript level. (f) Heatmap exhibits transcript level of genes in the integrin-based signature across low- and high-riskScore subpopulations from ICGC-LIRI-JP cohort.

**Figure 3:** The integrin-based signature excellently predicts HCC's OS outcome. (a) K-M curves depict the OS outcome of two subpopulations stratified by the median riskScore in TCGA-LIHC cohort. OS difference was inferred with log-rank test. (b) ROC curves validate the prediction efficacy of riskScore for OS at one, two together with three years in TCGA-LIHC cohort. (c) PCA plots demonstrate the discrepancy between low- and high-riskScore subpopulations from TCGA-LIHC cohort at the transcriptome level. (d) tSNE plots prove the discrepancy between low- and high-riskScore subpopulations from TCGA-LIHC cohort at the transcriptome level. (e) K-M curves show the OS outcome of two subpopulations stratified by the median riskScore in ICGC-LIRI-JP cohort. OS difference was computed utilizing log-rank test. (f) ROC curves validate the prediction efficacy of riskScore for OS at one, two together with three years in ICGC-LIRI-JP cohort. (g) PCA plots demonstrate the discrepancy between low- and high-riskScore subpopulations from ICGC-LIRI-JP cohort at the transcriptome level. (h) tSNE plots prove the discrepancy between low- and high-riskScore subpopulations from ICGC-LIRI-JP cohort at the transcriptome level.

**Figure 4:** The integrin-based signature is independent of routine clinicopathological parameters across TCGA-LIHC. (a, b) Forest diagram shows the associations of riskScore and routine clinicopathological parameters with OS outcome utilizing uni- and multivariate-cox regression approaches. (c–h) K-M curves of low- and high-riskScore subpopulations in diverse subgroups stratified by routine clinicopathological parameters.

**Figure 5:** Generation of an integrin-based signature- and stage-based nomogram into HCC clinical practice in TCGA-LIHC cohort. (a) The nomogram incorporating two independent risky factors (riskScore together with stage) for HCC. (b) ROC curves of OS at one, two together with three years. (c) The C-indices of various variables in short- and long-term OS outcomes. (d) Calibration plots of the nomogram for predicting the probability of OS at one, three, together with five years. (e–g) Decision curve analysis curves for inferring the bet benefits.

**Figure 6:** Selection of integrin-based signature-specific genes across TCGA-LIHC. (a) Gene dendrogram acquired through average linkage hierarchical clustering. The colored row below the dendrogram depicts the module assignment determined with dynamic tree cut approach. (b, c) Selection of the optimal soft threshold in accordance with scale independence together with mean connectivity. (d) Associations of coexpression modules with low- and high-riskScore specimens. Each module comprises correlation coefficient together with *p* value. (e) GO enrichment terms of genes in turquoise module. The length of the columns indicates the count of enriched genes. (f) KEGG pathways of genes in turquoise module. Red denotes high enrichment, and blue denotes low enrichment. The size of the dots represents the count of enriched genes. (g, h) GO enrichment terms together with KEGG pathways of genes in yellow module.

**Figure 7:** Interactions of the integrin-based signature with components within tumor microenvironment across TCGA-LIHC. (a) Heatmap illustrates the abundance of tumor microenvironment components in low- and high-riskScore subpopulations utilizing diverse computational approaches. (b) Associations of riskScore with the abundance of tumor microenvironment components. (c–i) Interactions of genes from the integrin-based signature and riskScore with the abundance of tumor microenvironment components computed through CIBERSORT, XCELL, CIBERSORT-ABS, QuantTIseq, MCPcounter, EPIC together with TIMER approaches. ^∗^*p* < 0.05; ^∗∗^*p* < 0.01; ^∗∗∗^*p* < 0.001.

**Figure 8:** The importance of LIMS2 from the integrin-based signature in HCC. (a) Assessment of the relative importance of genes in the integrin-based signature through adopting random-forest approach across TCGA-LIHC. (b) Transcript level of LIMS2 in low- and high-riskScore subpopulations across TCGA-LIHC. (c) Association of transcript level of LIMS2 with integrin-based signature-derived riskScore across TCGA-LIHC. (d, e) Immunohistochemical images of LIMS2 in normal and HCC tissues from the Human Protein Atlas. Bar, 200 *μ*m. (f) RT-PCR was applied to examine the expression of LIMS2 in HCC specimens and nontumor specimens. ^∗∗^*p* < 0.01.

## Data Availability

The data presented in this study are available from the corresponding authors on reasonable request.

## Abbreviations

HCC: Hepatocellular carcinoma
ECM: Extracellular matrix
LASSO: Least absolute shrinkage and selection operator
OS: Overall survival
K-M: Kaplan–Meier
AUC: Area under the receiver operating characteristic curve
C-index: Concordance index
WGCNA: Weighted gene coexpression network analysis
GO: Gene ontology
KEGG: Kyoto Encyclopedia of Genes and Genomes
FDR: False discovery rate.
